# Left Atrial Appendage Depth and Tachycardia Bradycardia Syndrome as Important Predictors of Left Atrial Appendage Thrombus in Patients with Nonvalvular Atrial Fibrillation

This article has been retracted.

**DOI:** 10.1155/2022/4632823

**Published:** 2022-03-30

**Authors:** Yinge He, Panpan Chen, Ziqiang Zhu, Junhua Sun, Yujie Zhao

**Affiliations:** Department of Cardiology, Zhengzhou No. 7 People's Hospital, No. 17, Jingnan Fifth Road, Economy and Technical Development Zone, Zhengzhou, Henan Province, 450000, China

## Abstract

**Background:**

Atrial fibrillation (AF) is the most common heart rhythm disorder that has been shown to be associated with a significant increase in stroke and systemic embolism risk. The left atrial appendage (LAA) is a finger-like extension originating from the left atrium; the formation of thrombus in LAA is the main reason of stroke and systemic embolism in patients with nonvalvular atrial fibrillation (NVAF). This study is aimed at finding out the risk of left atrial appendage thrombus (LAAT) in patients with nonvalvular atrial fibrillation (NVAF).

**Method:**

We retrospectively examined the clinic and left atrial computer tomography angiography (CTA) features of patients assessed in Zhengzhou No. 7 People's Hospital between January 2020 and January 2021 derivation. Student's *t*-test, chi-square test, receiver operating characteristics (ROC) curves, and logistic regression analysis were used to identify predictors of LAAT.

**Result:**

Of 480 patients included in the analysis, LAAT was found in approximately 9.2% of all patients. Univariate demographic predictors of LAAT included left atrium top and bottom diameter (LTD), left atrial appendage depth (LAAD), CHA2DS2-VASc, tachycardia bradycardia syndrome (TBS), and nonparoxysmal atrial fibrillation (PAF). In a multiple logistic regression analysis, the independent predictors of thrombus were LAAD > 23.45 mm (odds ratio: 4.216, 95% CI: 1.869-9.510, *P* = 0.001), TBS (odds ratio: 4.076, 95% CI: 1.655-10.038, *P* = 0.002), and non-PAF (odds ratio: 2.896, 95% CI: 1.183-7.094, *P* = 0.02).

**Conclusion:**

In NVAF patients with LAAT, evidence suggested that larger LAAD, non-PAF, and TBS present a high risk of LAAT. This is the first report demonstrating that the LAAD and TBS are associated with LAAT in patients with NVAF.

## 1. Introduction

Nonvalvular atrial fibrillation (NVAF) is independently associated with a four- to fivefold increased risk of ischemic stroke attributed to the thrombus from left atrium [1], and the number of AF patients is increasing annually [2]. Thrombus formation needs triad events [3, 4]: (1) endocardial damage or dysfunction and related structural abnormal changes, (2) abnormal blood stasis, and (3) abnormal haemostasis, platelets, and fibrinolysis; these variables are clearly evident in NVAF.

Left atrial appendage (LAA), a finger-like structure in the left atrium, has pectinate muscles with trabeculation leading to its uniqueness. LAA is the source of thrombus in more than 90% of the individuals with NVAF [5]. With the development of NVAF, the LAA develops mechanical dysfunction and fibroelastotic changes on the endocardial surface and this results in LAA remodeling and ultimately left atrial appendage thrombus (LAAT) [6–8]. A larger left atrial diameter, wider LAA orifice, and increased LAA depth indicate remodeling of the left atrial and LAA [9]; we measured the left atrium anteroposterior diameter (LAD), LTD, left atrial lateral diameter (LLD), maximum LAA ostium axis (max-LAAOA), minimum LAA ostium axis (min-LAAOA), and LAAD with CTA to compare the difference between the LAAT group and non-LAAT group.

TBS is characterized by prolonged sinus pause on the termination of atrial tachyarrhythmias. The association between AF and sick sinus syndrome has been long recognized and is thought to form the basis of TBS. AF promote structural abnormalities and electrical remodeling in the form of fibrosis in atrium and sinus node; this is considered to be the important mechanism for the occurrence of TBS in AF [10–12]. Based on the evidence, we hypothesize that AF patients with TBS have worse atrial fibrosis; this can lead to more serious atrial dysfunction and LAAT. In this study, TBS was included to explore whether it was a risk factor for LAAT.

## 2. Methods

### 2.1. Patient Population

The cohort included consecutive NVAF patients referred to Zhengzhou No. 7 People's Hospital between January 2020 and January 2021. All patients were first diagnosed with NVAF and did not receive anticoagulant therapy. All LAAT were detected on CTA.

Diagnosis of TBS was made by Holter electrocardiogram (ECG). All clinical data included gender, age, and CTA data (LAD, LTD, LLD, max-LAAOA, min-LAAOA, and LAAD). The history of disease included hypertension, diabetes, coronary heart disease (CHD), PAF, non-PAF, and massive regurgitation of mitral valve (MR of MV) assessed by transthoracic echocardiography.

All clinical, laboratory, and CTA data were obtained retrospectively from medical records.

### 2.2. Statistical Analysis

Continuous variables were expressed as the mean ± SD. Categorical variables were expressed as numbers and frequencies. Student's *t*-test was used to compare the differences in continuous variables. The chi-square test was used to compare the difference in incidence between the two groups. Logistic regression was used to assess risk markers. The ROC analysis was used to evaluate the predictive effect of the model on LAAT. All statistical tests were performed with SPSS 23.0 (developed by International Business Machines Corporation). *P* value of <0.05 was considered a signifificant statistical difference.

## 3. Results

### 3.1. Baseline Characteristics

Of the 480 patients who underwent CTA prior to therapy, we identified 37 patients with LAAT. All 480 patients were first diagnosed with atrial fibrillation and not took anticoagulation. 37 patients have LAAT (7.7%); compared with non-LAAT, LAAT patients were older and have a higher prevalence of hypertension, non-PAF, MR of MV and TBS; the CHA2DS2-VASc scores are higher too; larger LAD, LTD, LLD, max-LAAOA, min-LAAOA, and LAAD were also found in LAAT patients. There was no difference in gender, renal insufficiency, diabetes, and CHD (Table 1).

### 3.2. Predictors of LAAT

Multiple candidate clinical predictors and CTA measurements were assessed as univariate independent predictors for LAAT. The statistically significant univariate predictors of events were LTD, LAAD, CHA2DS2-VASc, TBS, and non-PAF (Table 2). Furthermore, we conducted ROC curve analysis to statistically significant parameters for LAAT prediction in patients with NVAF; the area under ROC curves (AUC) for LAAD was 0.735 (sensitivity: 75.7%, specificity: 74.9%, 95% CI: 0.66-0.82, *P* < 0.001). The AUC for LTD was 0.705 (sensitivity: 75.7%, specificity: 73.7%, 95% CI: 0.63-0.73, *P* < 0.001). The AUC for CHA2DS2-VASc was 0.736 (sensitivity: 10.8%, specificity: 96.4%, 95% CI: 0.63-0.73, *P* < 0.001) (Figure 1). The statistically significant multivariable predictors of events were LAAD > 23.45 mm (odds ratio: 4.216, 95% CI: 1.869-9.510, *P* = 0.001), TBS (odds ratio: 4.076, 95% CI: 1.655-10.038, *P* = 0.002), and non-PAF (odds ratio: 2.896, 95% CI: 1.183-7.094, *P* = 0.02) (Table 3).

## 4. Discussion

LAA possesses high compliance and forms a good reservoir for the blood in the heart to modulating the LA pressure [13]. LA strain caused by NVAF can directly measure LAA remodeling which manifests itself as enlargement of LAA orifice area and volume [14–19], and remodeling was associated with LAAT [20–25]. Remodeling means not only larger size but also greater endocardial thickening with fibrous tissue making a decreased velocity in LAA, further affecting LAA emptying; these may play a role in LAA thrombus formation in NVAF [19, 22–29]. LAA depths were also associated with increased LAAT in our study. Our findings support the notion that the remodeling of LAA depth is involved in the chain of events leading from NVAF to LAAT. Therefore, any direction of the LAA remodeling will result in LAAT.

Another attributing factor is TBS. A proportion of AF patients have TBS. Prolonged sinus pauses can be observed in AF patients; that is a condition known as TBS [30]. Sinus node (SN) dysfunction is the main reason of TBS; SN remodeling caused by atrial tachyarrhythmia, including AF, leads to reversible SN dysfunction [31, 32]. AF can lead to anatomical and electrophysiological remodeling within the SN and surrounding atrial tissue that prompts and accelerates the development of SN dysfunction [33]; fibrosis is a key aspect of remodeling which serves to slow conduction and cause atrial contractile dysfunction [34]. In AF patients, LAA remodeling occurs in both left and right atrial appendages, but more severe endocardial changes were found in the LAA than that in the right atrial appendage (RAA) [35]; TBS means serious RAA remodeling; there may also be severe remodeling in LAA that leads to LAAT. LA blood emptying benefits from active atrial contraction and passive ventricular diastolic emptying, which is also the decisive factor of LAA emptying [27], TBS occurs, and the ventricle stops contracting and diastolic, causing further blood stasis in the atria which has lost the ability to contract; those contribute to LAAT. Our results found that patients with non-PAF had a higher risk of LAAT.

Patients with non-PAF had a significant higher risk of LAAT; these findings are consistent with the study before [36–38]. The major difference between paroxysmal AF and non-PAF is whether AF is sustained. Atrial substrate is the most important factor to sustain AF that means atrial remodeling [39, 40]. Remodeling results in severe fibrosis of LA and LAA, which leads to systolic dysfunction and decreased LAA flow velocity as compared with PAF [38]. This makes non-PAF more prone to LAA. This is consistent with our findings.

## 5. Limitations

Our study had several limitations. First, the study was retrospect analysis. Second, we did not analyze the history of peripheral embolism because the data were incomplete. Most patients with acute cerebral infarction are treated in the department of neurology; for some of those patients, screening for atrial fibrillation was neglected. Third, LAAT measured by CTA does not have 100% sensitivity in detecting LAAT.

## 6. Conclusion

There are many factors that impact on thromboembolic events in NVAF patients. This study suggests that large LAAD, non-PAF, and TBS may present a high risk group of LAAT.

## Figures and Tables

**Figure 1:** ROC curve for LAAD, LTD, and CHA2DS2-VASc score. LAAD: left atrial appendage depth; LTD: left atrium top and bottom diameter.

**Table 1:** Demographic and clinical data of patients.

	LAAT *N* = 37 (%)	Non-LAAT *N* = 443 (%)	*P* value
Male	18 (48.6)	280 (63.2)	0.111
Age (≧75)	13 (35.1)	71 (16)	0.006
Renal insufficiency	5 (13.5)	29 (6)	0.169
Diabetes	13 (35.1)	105 (23.7)	0.162
Hypertension	25 (67.6)	207 (46.7)	0.017
Non-PAF	30 (81)	222 (50.1)	<0.001
CHD	21 (56.8)	198 (44.7)	0.172
CHA2DS2-VASc	4.46 ± 1.71	2.86 ± 1.88	<0.001
MR of MV	15 (40.5)	109 (24.6)	0.049
TBS	9 (24.3)	28 (6.3)	0.003
LAD	55.84 ± 8.37	48.35 ± 9.63	<0.001
LTD	66.14 ± 7.88	60.23 ± 7.92	<0.001
LLD	81.86 ± 8.98	75.43 ± 10.17	<0.001
Max-LAAOA	30.12 ± 5.49	28.00 ± 5.42	0.023
Min-LAAOA	20.84 ± 5.07	24.30 ± 5.13	<0.001
LAAD	26.21 ± 4.52	22.36 ± 4.46	<0.001

LAAT: left atrial appendage thrombus; non-PAF: nonparoxysmal atrial fibrillation; CHD: coronary heart disease; MR of MV: massive regurgitation of mitral valve; TBS: tachycardia bradycardia syndrome; LAD: left atrium anteroposterior diameter; LTD: left atrium top and bottom diameter; LLD: left atrial lateral diameter; max-LAAOA: maximum left atrial appendage ostium axis; min-LAAOA: minimum left atrial appendage ostium axis; LAAD: left atrial appendage depth.

**Table 2:** Binary logistic regression analysis for risk markers.

	OR	95% CI	*P* value
Non-PAF	3.30	1.252-8.710	0.016
CHA2DS2-VASc	1.421	1.110-1.819	0.005
LTD	1.070	1.009-1.135	0.025
LAAD	1.155	1.048-1.272	0.004
TBS	0.165	0.062-0.442	<0.001

non-PAF: nonparoxysmal atrial fibrillation; LTD: left atrium top and bottom diameter; LAAD: left atrial appendage depth; TBS: tachycardia bradycardia syndrome.

**Table 3:** Multivariate logistic regression analysis for risk markers.

	OR	95% CI	*P* value
LAAD > 23.45 mm	4.216	1.869-9.510	0.001
Non-PAF	2.896	1.183-7.094	0.02
TBS	4.076	1.655-10.038	0.002

LAAD: left atrial appendage depth; non-PAF: nonparoxysmal atrial fibrillation; TBS: tachycardia bradycardia syndrome.

## Data Availability

The data used to support the findings of this study are available from the corresponding author upon request.
